# Ultrasound-Guided Median Nerve Electrical Stimulation to Promote Upper Limb Function Recovery after Stroke

**DOI:** 10.1155/2022/3590057

**Published:** 2022-07-14

**Authors:** Rui Li, Jingyi Lu, Meiqi Wang, Ping Zhang, Hongmei Fang, Kunli Yang, Liuyan Wang, Jianlin Zhuang, Zhihe Tian, Jianming Yang, Qing Luo, Zhufen Yang, Kai Ling Chin

**Affiliations:** ^1^Department of Rehabilitation Medicine, The Second People's Hospital of Kunming, Rehabilitation Hospital, Kunming University, Kunming 650204, China; ^2^Department of Biomedical Sciences, Faculty of Medicine & Health Sciences, Universiti Malaysia Sabah, Kota Kinabalu 88400, Sabah, Malaysia

## Abstract

Peripheral electrical nerve stimulation enhances hand function during stroke rehabilitation. Here, we proposed a percutaneous direct median nerve stimulation guided by ultrasound (ultrasound‐guided median nerve electrical stimulation, UG-MNES) and evaluated its feasibility and effectiveness in the treatment of stroke patients with upper limb extremity impairments. Sixty-three stroke patients (2-3 months of onset) were randomly divided into control and UG-MNES groups. Both groups received routine rehabilitation and the UG-MNES group received an additional ultrasound-guided electrical stimulation of the median nerve at 2 Hz, 0.2 ms pulse-width for 20 minutes with gradual intensity enhancement. The Fugl-Meyer Assessment for upper extremity motor function (FMA-UE) was used as the primary outcome. The secondary outcomes were the Functional Test for the Hemiplegic Upper Extremity (FTHUE-HK), Hand Function Rating Scale, Brunnstrom Stages, and Barthel Index scores for motor and daily functions. All the participants completed the trial without any side effects or adverse events during the intervention. After 4 weeks of intervention, the functions of the upper limbs on the hemiplegic side in both groups achieved significant recovery. Compared to the control group, all evaluation indices used in this trial were improved significantly in the UG-MNES group after 2 and 4 weeks of intervention; particularly, the first intervention of UG-MNES immediately improved all the assessment items significantly. In conclusion, the UG-MNES is a safe and feasible treatment for stroke patients with upper limb extremity impairments and could significantly improve the motor function of the affected upper limb, especially in the first intervention. The UG-MNES could be an effective alternative intervention for stroke with upper limb extremity impairments.

## 1. Introduction

Stroke is the leading cause of death and long-term disability around the world. Although the application of developing medical technology decreases the rates of stroke mortality significantly, most survivors still suffer from neurological deficits such as motor, memory, and cognitive dysfunctions, which results in an immense economic burden on society and families [1, 2]. The upper limb extremity impairments are the most frequent dysfunction following stroke; that is, more than 70% of stroke patients suffer from the paretic arm. Only 5–20% of the patients achieve complete functional recovery after 6 months of onset [3–5]. The impaired upper limb severely limits the independent daily activities of stroke patients. Thus, restoration of upper limb function is vital to the treatment and rehabilitation of stroke. To date, the commonly applied rehabilitation techniques such as classical physiotherapy and impairment-oriented training are limited by efficacy [6–8]. Consequently, it is urgent to establish and explore some efficacious treatments for improving upper limb functional recovery after cerebral ischemia.

Recently, the electrical stimulation applied to the brain and peripheral nervous system has been recognized as a promising treatment for functional recovery after stroke. The transcranial direct current stimulation (tDCS) is a noninvasive brain stimulation technique that can initiate a long-term potentiation or long-term depression and then induce the cortical plasticity and improve the nerve functional restoration of the upper limb motor [9], movement planning and preparation [10], and hemispatial neglect [11]. The clinical effects of tDCS depend on the injured site and the stimulus parameters, and it is difficult to achieve precision function therapy, such as the promotion of upper limb function. The peripheral electrical stimulation has been confirmed as a safe and effective treatment for functional recovery after stroke by stimulating the peripheral neuromuscular system and inducing the cortical plasticity [12, 13]. Currently, the peripheral electrical stimulation includes the functional electrical stimulation (FES), the transcutaneous or neuromuscular electrical stimulation (TENS or NMES), and the transcutaneous electrical acupoint stimulation (TEAS) which combined the meridian theory of traditional Chinese medicine and repetitive sensory stimulation (RSS). These noninvasion peripheral electrical stimulation therapies can stimulate the senses, increase muscle power and movement function, and decrease limb spasticity through various stimulus currents and protocols [14, 15]. Meanwhile, peripheral electrical stimulation-induced brain plasticity contributes to the long-term functional improvement [12, 16].

The median nerve mixed with sensory and motor fibers is a primary important nerve of the hand. It innervates the flexor-pronator muscles in the forearm and most muscle groups in the hand and controls flexion of the wrist, abduction of the thumb, and flexion of the fingers [17]. The electrical stimulation on the area of the median nerve (MNES, usually located on the wrist above the median nerve) increases pinch strength [18] and facilitates the effects of rehabilitation training [19, 20] after stroke. However, these cutaneous MNES stimulate both the median nerve and other tissues. It is difficult to target the median nerve specifically at the same time and determine the optimal stimulus parameters. Implanted electrodes can target specific nerves and reduce the current required to stimulate the nerve. Recently, using a rat model of experimental stroke, the group of Tsai et al. [21] observed that direct median nerve stimulation significantly improved both the motor skills and sensory recovery in the impaired forelimb. Also, the direct MNES promoted the neural plasticity in the cervical spinal cord detected by axonal tracing of biotinylated dextran amine. However, implanted direct nerve stimulation needs an operation and might cause some problems such as long-term biological compatibility and nerve damage. Ultrasound-guided nerve electrical stimulation can target the specific nerve through a percutaneous fine-needle electrode under ultrasound guidance. The ultrasound-guided nerve electrical stimulation has been used for the relief of postamputation pain [22–24]. However, the feasibility and effectiveness of ultrasound-guided nerve electrical stimulation in the treatment of stroke remain unknown.

The recovery of upper limb function after stroke is a difficult task in rehabilitation. In this study, our team innovatively proposed and applied the musculoskeletal ultrasound intervention technique in clinical practice, combining the nerve electrical stimulation technique with the ultrasound technique. The ultrasound-guided median nerve electrical stimulation (UG-MNES) technique was used to treat the upper limb dysfunction after stroke. The treatment significantly improved the upper limb motor function in the immediate poststroke period which is worthy of clinical promotion and application.

## 2. Materials and Methods

### 2.1. Study Design

This study adopted an assessor-blinded, randomized controlled design. All subjects were randomized to control with conventional rehabilitation (control group) and UG-MNES group. A separate investigator who was blind to experiment design was responsible for the functional assessments. The experimental procedure was approved by the Human Ethics Committee of the Second People's Hospital of Kunming (ethical approval no. 2019–01).

### 2.2. Participants

A total of 63 stroke patients with upper extremity hypotonia were recruited from the Department of Rehabilitation in the Second People's Hospital of Kunming. The inclusion criteria were as follows: (1) meeting the diagnostic criteria of cerebral stroke and confirmed by brain computed tomography (CT) or magnetic resonance imaging (MRI) examination; (2) first-ever ischemic or hemorrhagic stroke and during 2-3 months of onset; (3) Brunnstrom Stages of 1-2 in upper limb; and (4) stable vital signs without severe cognitive impairment. Exclusion criteria were as follows: (1) unstable or uncontrollable systemic diseases; (2) hemiplegic upper limb skin ulcer and inflammation; and (3) severe emotional, visual, and cognitive impairments.

### 2.3. Procedures

All participants in the study voluntarily signed the written informed consent form. Before the study, basic information, including age, sex, lesion side of the brain, stroke type, and duration after stroke onset, was recorded. The subjects who met the criteria were randomly divided into UG-MNES and control groups. All the participants in both groups received routine rehabilitation, including hemiplegia exercise training therapy, occupational therapy, physical factor therapy, or traditional therapy, according to the actual situation of the patients. The frequency of rehabilitation is 30 to 40 minutes, once a day, 5 to 6 times a week, for a total of 4 weeks. The intensity is appropriate for the patients without any obvious sense of fatigue. In addition to routine rehabilitation, the UG-MNES group received invasive percutaneous electrical stimulation of the median nerve under ultrasound guidance. The electrical stimulation of the median nerve was stimulated once a week for a total of 4 weeks, each time for 20 minutes with a total of 4 times' stimulation. The control group was evaluated before treatment and 2 and 4 weeks after treatment, while the UG-MNES group was evaluated before and immediately after treatment at 1, 2, 3, and 4 weeks. Assessments were conducted including Fugl-Meyer Assessment for upper extremity (FMA-UE), Functional Test for the Hemiplegic Upper Extremity (FTHUE-HK), Hand Function Rating Scale, Brunnstrom Stages, and Barthel Index scores (Figure 1).

### 2.4. Ultrasound‐Guided Median Nerve Electrical Stimulation

The detailed procedures of median nerve electrical stimulation guided by ultrasound were as follows. The patient's forearm is placed in a posteriorly rotated position on a treatment pillow. A disposable electrical stimulation needle (with 0.5 mm diameter and 50 mm long) was used at 7–10 cm from the forearm of the affected side to the transverse striae of the wrist under the short-axis section. Depending on the length of the patient's arm, the location of the puncture point was selected in which the median nerve penetrates between the deep finger flexors and the superficial finger flexors, where the median nerve is superficial, and the image obtained under ultrasound guidance is the clearest. The short-axial plane of ultrasound was selected to allow the needle to be as perpendicular to the nerve trunk as possible to maximize the intensity of the current field. The needle was inserted in the plane to avoid the blood vessel tendon until the tip was found close to the nerve sheath membrane under ultrasound. The end of the needle core was connected to the peripheral nerve electrical stimulator (model SY-708A) (Figure 2). A bidirectional rectangular wave of an internal model was adopted with a frequency of 2 Hz and a pulse width of 0.2 ms. The stimulus current was adjusted to 1.0 mA for 5 minutes to trigger the thumb and forefinger palm and flexion movement. Then, the amount of stimulation was increased to 1.5 mA for 10 minutes. The amount of stimulation was increased again to 1.8 mA for 5 minutes and the needle was removed. The comprehensive evaluation of hemiplegic upper limb function on the hemiplegic side was performed before and immediately after treatment at 1, 2, 3, and 4 weeks, for a total of 8 assessments.

### 2.5. The Primary Outcome Assessment

The Fugl-Meyer Assessment of upper extremity (FMA-UE) was used as the primary outcome. The FMA-UE is a well-recognized and recommended observational measure of upper limb impairments. The FMA-UE assessment includes 7 parts, that is, (1) upper limb reflex activity, (2) flexor joint movement, (3) extensor joint movement, (4) isolated movement, (5) normal reflex activity, (6) wrist stability, and (7) finger movement. The maximum score of motor function of FMA-UE is 66.

### 2.6. The Secondary Outcome Assessments

The assessment of Functional Test for the Hemiplegic Upper Extremity (FTHUE-HK), Hand Function Rating Scale, Brunnstrom Stages, and Barthel Index scores were used as the secondary outcomes.

#### 2.6.1. FTHUE-HK

The assessment of Functional Test for the Hemiplegic Upper Extremity (FTHUE-HK) was as follows: Level 1: no reaction; Level 2: (A) associated reaction, (B) the affected hand was placed on the ipsilateral thigh; Level 3: (C) lift the affected arm while tucking in the affected side clothes into the pants with healthy hands, (D) carry a bag weighing 1 kg (lasts for 15 seconds); Level 4: (E) stabilize the bottle cap (open the bottle cap with the healthy hand and hold the cup with the affected hand), (F) fix one end of the towel with the affected hand and wring the wet towel dry (twist the healthy hand twice); Level 5: (G) pick up and move small pieces of wooden blocks, (H) eat with a spoon; Level 6: (I) lift a box, (J) drink water from a plastic cup; Level 7: (K) use a key to open a lock, (L1) manipulating chopsticks (dominant hand), (L2) manipulating clamps (nondominant hand).

#### 2.6.2. Hand Function Rating Scale

It includes the evaluation of 5 practical prescribed movements: cutting with scissors, taking coins out of wallets, opening umbrellas, cutting fingernails, and fastening buttons on the sleeves with six-level of assessments, that is, lost hand function: cannot complete all the five actions; assistive hand D: five actions can only complete one; assistive hand C: five actions can only complete two; assistive hand B: five actions can complete three; assistive hand A: five actions can complete four; practical hand: complete all five actions.

#### 2.6.3. Brunnstrom Stages

The upper extremity is primarily evaluated in six stages, going from involuntary movement to increase muscle tone to common movement, dissociative movement, and later more dissociative movement, culminating in speed and coordination close to normal movement.

#### 2.6.4. Barthel Index

It consists of ten items: eating, transferring from wheelchair to bed, grooming, going to the bathroom, taking a bath, walking, climbing up and down stairs, wearing and undressing, bowel control, and bladder control.

### 2.7. Data Analysis

Data analysis was conducted using the Statistical Package for the Social Sciences (SPSS) version 25.0. Shapiro-Wilk test was used to examine the normal distribution of the underlying model assumptions. Categorical variables were expressed as absolute (*n*) and percentage (%), while continuous variables were expressed as mean ± standard deviation or median (1st–3rd quartiles) [M (P25–P75)], depending on the data distribution. Baseline characteristics for categorical variables between groups (i.e., gender and stroke type) were compared using the chi-square test or Fisher's exact test. Baseline characteristics for continuous variables between groups were examined with the Mann-Whitney *U* test (i.e., duration of disease and NIHSS score) and *t-*test (i.e., age). The Wilcoxon signed rank-sum test was used to compare FMA-UE, FTHUE-HK, Hand Function Rating Scale, Brunnstrom Stage, and Barthel Index scores between the two groups before and after 2 and 4 weeks of treatment. The Wilcoxon rank-sum test was used to test for differences between before and immediately after intervention in the UG-MNES group. The statistical level of significance was *p* < 0.05.

## 3. Results

### 3.1. Comparison of General Data between the Two Groups

The patients who met the inclusion criteria were randomly divided into the control group (*n* = 31) and the UG-MNES group (*n* = 32). The mean age of the control group was 56.39 ± 2.11, and the mean age of the UG-MNES group was 54.5 ± 2.12. There was no significant difference in age and gender between the two groups (*p* > 0.05). There was no difference in time after stroke and stroke type (cerebral hemorrhage and cerebral infarction) between the groups (*p* > 0.05). There was no significant difference in neurological deficit scores between the groups (*p* > 0.05). The general data of all participants are summarized in Table 1.

### 3.2. The Median Nerve Stimulation Group and the Routine Rehabilitation Group Improve the Function of the Upper Limbs of Hemiplegic Patients with Stroke

Before treatment, there was no significant difference in upper limb motor function, Brunnstrom Stage, and activities of daily living between the control and UG-MNES groups (*p* > 0.05). After 2 and 4 weeks of treatment, the motor function of the upper limbs and activities of daily living of hemiplegic patients with stroke had a significant improvement in both the control and UG-MNES groups (*p* < 0.05).

The Fugl-Meyer motor function score of the upper limbs in the UG-MNES group was higher than that in the control group (*p* < 0.01) at 2 weeks of treatment and *p* < 0.05 at 4 weeks of treatment (Table 2 and Figure 3).

Compared to the control group, the median nerve stimulation significantly enhanced the motor impairment of the upper limb assessed by FTHUE-HK and Hand Function Rating Scale at 2 and 4 weeks of treatment. The hand function classification of hemiplegia in the UG-MNES group was mainly Grade 3, while in the control group was mostly Grade 2 (*p* < 0.01) (Tables 3 and 4 and Figures 4 and 5).

Similarly, after 4 weeks of trial, the Brunnstrom motor stages of the upper limbs on the hemiplegic side in the UG-MNES group had reached Stages 3 and 4, while those in the control group were mostly in Stages 2 and 3. There was a significant difference in Brunnstrom Stages between the two groups (*p* < 0.01) (*P* < 0.01)(Table 5 and Figure 6).

The Barthel Index for activities of daily living in the UG-MNES group was slightly higher than that in the control group at 2 and 4 weeks of treatment (*p* < 0.01)(*P* < 0.01) (Table 6 and Figure 7). This result indicated that improved hand function in the UG-MNES group had contributed to the improved activities of daily living function.

### 3.3. Ultrasound-Guided Electrical Stimulation of the Median Nerve Immediately Improved the Function of the Upper Extremity on the Hemiplegic Side

In this trial of 4 consecutive weeks, the patients in the UG-MNES group received 4 ultrasound-guided electrical stimulation (once a week). The upper limb functions on the hemiplegic side were assessed before and immediately after each stimulus. The results showed that ultrasound-guided electrical stimulation of the median nerve immediately improved the Fugl-Meyer Assessment of the upper extremity motor function on the hemiplegic side on the first, third, and fourth intervention. In particular, the first intervention immediately improved all the assessment items including FMA-UE, FTHUE-HK, Brunnstrom Stages, Hand Function Rating Scale, and Barthel Index scores. However, the immediate improvement effect on motor and daily functions did not last into the second, third, and fourth week. These results indicated that the ultrasound-guided electrical stimulation of the median nerve mainly improved the gross function of the upper extremity (Table 7).

## 4. Discussion

In this study, we proposed a percutaneous direct median nerve stimulation guided by ultrasound (UG-MNES) and evaluated its feasibility and effectiveness in the treatment of stroke patients with upper limb extremity impairments. The UG-MNES stimulates the median nerve directly without surgical incision through the insertion of a lead under ultrasound guidance. All patients who participated in this study completed the intervention without any adverse events and side effects, proving that UG-MNES was safe and feasible in treatment for stroke patients with upper limb extremity impairments. This study confirmed that UG-MNES could improve the function of the affected upper limb; in particular the first intervention immediately improved all assessment items including FMA-UE, FTHUE-HK, Brunnstrom Stages, Hand Function Scale, and Barthel Index. These results indicated that the UG-MNES could be an effective intervention for stroke patients with upper limb extremity impairments.

Stroke damages the important region in the brain, such as the motor cortex and sensory cortex, destroys the neural network connection, and results in the loss of sensory and motor function in the affected extremity. The structural damage during stroke initially occurs only in the brain and the peripheral nervous system and its target organs such as skeletal muscle are structurally intact. The disconnected network in the brain results in the denervation of skeletal muscle fiber and further leads to various functional disorders. The persistent lack of nerve stimulation leads to the structural and functional abnormality of the neuromuscular junction (NMJ) and the atrophy in denervated muscle. The disconnected network in the brain and the abnormality in NMJ together contribute to various dysfunctions after stroke and increase the difficulty of rehabilitation treatment during the sequela stage of stroke. Thus, the targets for poststroke treatment need to focus on the neural plasticity of the brain and the functional reconstruction between the nervous system and the muscular [25, 26].

The nervous system is complicated and closed, and the peripheral stimulation can promote the plasticity of the center neural system and improve the recovery of neural function, such as repetitive sensory stimulation (RSS), repetitive somatosensory electrical stimulation (SES), electrical stimulation of peripheral nerves, and passive rehabilitation training [27, 28]. RSS facilitates the neuroplastic processes in cortical areas that represent the site of sensory stimulation and improve sensorimotor performances (light-touch, tactile discrimination, and proprioception) through altering cortical maps and cortical excitability [29, 30]. In a clinical study of SES used for the treatment of acquired brain injury and distal upper limb motor impairments, Adelyn et al. found that SES in median and ulnar nerves induced cortical oscillations detected by electroencephalograph (EEG) and identified typical electrophysiological biomarkers [ipsilesional motor theta (4.8–7.9 Hz) and alpha (8.8–11.7 Hz)] which were significantly correlated with finger fractionation improvements [31]. Using functional near-infrared spectroscopy (fNIRS), Huo et al. [32] observed that median nerve electrical stimulation triggered sensorimotor stimulations of the affected hand and induced functional reorganization of distant cortical areas after stroke. These reports confirmed that transcutaneous peripheral electrical nerve stimulation could induce neuroplasticity in the sensorimotor cortex of the brain. In addition, the functional electrical stimulation (FES) triggered by surface electromyography in the uninjured limb or cortical signals was able to stimulate voluntary muscle activity, decrease spasticity in the affected limb, and improve the restoration of motion function [33–35]. In contrast to transcutaneous peripheral electrical nerve stimulation described above, the FES stimulated the paretic muscles, maintaining and improving their activity [36]. Some studies indicated that FES is more effective than TENS at improving gait speed after stroke [37].

Although the noninvasive peripheral electrical nerve stimulation enhanced hand function during stroke rehabilitation through neural plasticity in the brain and the maintenance of NMJ, The transcutaneous devices also stimulated some nontargeted nerves and muscles and are difficult to target the deeper nerves and muscles. Direct electrical nerve stimulation can target specific nerves and duration while reducing nontargeted nerve activation [21]. Because the median nerve carries both sensory and motor nerve fibers, the direct electrical stimulation of the median nerve could activate NMJ and paretic muscles through the motor nerve fibers and improve the hand function immediately. Meanwhile, the direct electrical stimulation on median nerve could enhance cortical excitability and induce neural plasticity in the brain, which led to long-term functional improvement [38, 39]. In this study, we observed that the first week of direct electrical stimulation for 20 minutes significantly promoted the hand function, but the improvement tended to decline in the subsequent interventions. This might be due to the limit of the activity of NMJ and paretic muscles. Additionally, the advantage of ultrasound-guided median nerve electrical stimulation is almost noninvasive, easy to operate, and safe.

The study has some limitations. Firstly, although to our knowledge we first proposed the direct median nerve stimulation guided by ultrasound (UG-MNES) and observed the effectiveness for the treatment of stroke, we need to compare the effects with noninvasive peripheral electrical nerve stimulation such as RSS and FES. Secondly, it is necessary to apply some objective evaluation indices such as functional magnetic resonance imaging (fMRI) and near-infrared spectroscopy to all the outcomes from the assessment scale. Thirdly, the optimal intervention plan of UG-MNES needs to be further explored, including intensity, duration, and interval time. Lastly, the undergoing cellular mechanism needs to be investigated.

## 5. Conclusion

In conclusion, the UG-MNES is safe and feasible in the treatment of stroke patients with upper limb extremity impairments and could improve the function of the affected upper limb; in particular the first intervention immediately improved all assessment items. The clinical application of the UG-MNES technique for the treatment of upper limb dysfunction in stroke was effective, but the effect was maintained for a short period of time, with significant immediate effect and no significant long-term effect, which may be related to the loss of nerve in the upper limb after stroke. Thus, there is a need to investigate its mechanism of action. At present, we adopted the model of gradual intensity enhancement, and the parameter selection is based on the evoked action and patient tolerable intensity. The parameter selection of electrical stimulation needs to be further optimized and explored to finally form a new treatment method for upper limb dysfunction in stroke. Our results indicated that the UG-MNES could be an effective rehabilitation intervention for stroke with upper limb extremity impairments.

## Figures and Tables

**Figure 1:** Flowchart of the study.

**Figure 2:** Median nerve electrical stimulation under ultrasound: (a) median nerve imaging of longitudinal section, (b) median nerve imaging of transection, (c) the ultrasound-guided median nerve electrical stimulation, and (d) UG-MNES ultrasound image. The white arrow points to the median nerve and the yellow arrow points to the electrical stimulation needle.

**Figure 3:** UG-MNES promoted the FMA-UE scores.

**Figure 4:** UG-MNES promoted the FTHUE-HK scores.

**Figure 5:** UG-MNES promoted the Hand Function Rating Scale.

**Figure 6:** UG-MNES improved the Brunnstrom Stages.

**Figure 7:** UG-MNES improved the Barthel Index.

**Table 1:** Demographic and clinical characteristics of subjects.

Team		Control group (*n* = 31)	Experimental group (*n* = 32)	*p*
Age (years)		56.39 ± 2.11	54.5 ± 2.12	0.531

Gender (*n*, %)	M	17 (54.8)	17 (53.1)	0.892
	F	14 (45.2)	15 (46.9)	

Time after stroke (months) M (P25, P75)		2 (1, 3)	2 (1, 3)	0.736

Stroke type (*n*, %)	CI	17 (54.8)	10 (31.25)	0.061
	CH	14 (45.2)	22 (68.75)	

NIHSS score M (P25, P75)		10 (7, 13)	8 (6.25, 9)	0.061

M: male; F: female; CI: cerebral ischemia; CH: cerebral hemorrhage.

**Table 2:** Comparison of FMA-UE scores in the two groups, M (P25, P75).

Team	Before	2 weeks	4 weeks
Control group (*n* = 31)	6 (4, 9)	13 (8, 17)	20 (10, 26)
Experimental group (*n* = 32)	6.5 (4, 9)	19 (16, 22)	26 (19.25, 30)
*Z*	4.42	3.21	2.225
*P* value	0.659	0.001	0.026

**Table 3:** Comparison of FTHUE-HK in the two groups, M (P25, P755).

Team	Before	2 weeks	4 weeks
Control group (*n* = 31)	1 (1, 2)	3 (2, 3)	3 (3, 4)
Experimental group (*n* = 32)	1 (1, 2)	3 (3, 4)	4 (4, 4.75)
*Z*	0.99	2.219	2.687
*P* value	0.32	0.027	0.007

**Table 4:** Comparison of Hand Function Rating Scale in the two groups, M (P25, P75).

Team	Before	2 weeks	4 weeks
Control group (*n* = 31)	1 (1, 2)	2 (2, 3)	2 (2, 3)
Experimental group (*n* = 32)	1 (1, 2)	3 (2, 3)	3 (3, 3)
*Z*	0.079	2.818	4.291
*P* value	0.937	0.005	<0.001

**Table 5:** Comparison of Brunnstrom Stages in the two groups, M (P25, P75).

Team	Before	2 weeks	4 weeks

Control group (*n* = 31)	2 (1, 2)	2 (2, 3)	2 (2, 3)
Experimental group (*n* = 32)	2 (1, 2)	3 (2, 3)	3 (2.25, 4)
*Z*	0.366	2.099	3.240
*P* value	0.714	0.036	0.001

**Table 6:** Comparison of Barthel Index in the two groups, M (P25, P75).

Team	Before	2 weeks	4 weeks
Control group (*n* = 31)	20 (15, 25)	35 (30, 40)	40 (35, 45)
Experimental group (*n* = 32)	20 (15, 25)	40 (35, 45)	45 (40, 55)
*Z*	0.691	2.721	2.690
*P* value	0.490	0.007	0.007

**Table 7:** Comprehensive function assessment of the affected upper limb before and immediately after median nerve electrical stimulation, M (P25, P75).

Outcomes	1 week before immediately	*p* value*P*	2 weeks before immediately	*p* value*P*	3 weeks before immediately	*Pp* value	4 weeks before immediately	*p* value*P*
FMA-UE	6.5 (4, 9)	*p* < 0.0001*P* < 0.0001	11 (8, 13.75)	0.243	19 (16, 22)	0.039	20 (16, 23.75)	0.004
	12 (12, 14.75)		11 (10, 13.75)		20 (16, 23.75)		28 (21.25, 32)	
FTHUE-HK	1 (1, 2)	*p* < 0.0001*P* < 0.0001	3 (2, 3)	0.068	3 (3, 4)	0.035	4 (4, 4.75)	0.129
	3 (2, 3)		3 (3, 3)		4 (3, 4)		4 (4, 5)	
Brunnstrom	2 (1, 2)	*p* < 0.0001*P* < 0.0001	2 (2, 2)	0.140	2 (2, 3)	0.102	3 (2.25, 4)	0.705
	3 (3, 3)		2 (2, 3)		3 (2, 3)		3 (3, 3)	
Hand Function	1 (1, 2)	*p* < 0.0001*P* < 0.0001	2 (2, 3)	0.138	2 (2, 3)	0.417	3 (3, 3)	0.152
	3 (2, 3)		3 (2, 3)		3 (2, 3)		3 (3, 4)	
Barthel Index	20 (15, 25)	*p* < 0.0001*P* < 0.0001	32.5 (25, 40)	0.003	40 (35, 45)	0.252	40 (35, 50)	0.104
	35 (31.25, 47.5)		35 (30, 40)		40 (40, 45)		47.5 (40, 55)	

FMA-UE: Fugl-Meyer Assessment of upper extremity, FTHUE-HK: Functional Test for the Hemiplegic Upper Extremity. *Pp* value: before the intervention *versus* after the intervention immediately.

## Data Availability

The data used to support the findings of this study are available within the article.
